The article "Innovation Clustering Analysis of Accurate Support Path for CSE under the Environment of Big Data" was retracted in 2023. Reasons: signs of a paper mill; suspected computer-generated content; unreliable results or conclusions; concerns about the data.

# Innovation Clustering Analysis of Accurate Support Path for CSE under the Environment of Big Data

**DOI:** 10.1155/2022/9706200

**Published:** 2022-09-29

**Authors:** Jianhai Hu

**Affiliations:** School of Digital Commerce (School of Cross-Border E-Commerce & Entreprenurship), Zhejiang Yue Xiu University, Shaoxing, 312000 Zhejiang, China

## Abstract

Facing the severe employment situation and social environment, the employment of college students has become a very important issue. The big data analysis plays a positive role in entrepreneurship, which can not only improve the success rate of entrepreneurial path selection, but also accumulate a lot of innovative practical experience for college students. Based on the importance of big data technology for entrepreneurial path, this paper proposes an innovative model of accurate support path for college students' entrepreneurship (CSE), in which the *K*-means algorithm is applied to the analysis of entrepreneurial support path. Finally, this paper makes an experimental analysis on the model, and the results show that *K*-means can greatly reduce the computational complexity of the algorithm, and the precision, recall, and F parameter of the model can be effectively improved. The model is of great significance in improving the feasibility of college students' entrepreneurial support policies.

## 1. Introduction

In recent year, some enterprises reduce the recruitment demand to reduce the cost, which leads to the unsatisfactory employment situation of college students [1]. Facing the current severe employment situation and social environment, college students' employment has become a very important issue, so it is of practical significance to support and solve the current employment problems. In recent years, it is more difficult for college students to find jobs, and the innovation and entrepreneurship can alleviate the employment problem of college students [2]. Based on the importance of entrepreneurship in solving the employment problem, the local government has strengthened the importance of innovation and entrepreneurship. The big data analysis is one of the important performance characteristics of big data technology, which plays an obvious role in the innovation and entrepreneurship [3, 4]. The big data analysis can bring more accurate judgment to college students' entrepreneurial path selection, which plays a positive role in social development and market economy. By mining potential entrepreneurial information resources, the big data analysis can help college students grasp better entrepreneurial opportunities. The application of big data analysis in precise entrepreneurship support can not only improve the feasibility of college students' entrepreneurship support policy, but also improve the purpose of policy.

In recent year, scholars have carried out a series of studies on the precise support for college students' entrepreneurship. At present, the research on the entrepreneurship policy of college students mainly focuses on the preferential policies, which are the venture capital support, the entrepreneurship education, the entrepreneurship service, and the entrepreneurial environment. According to the different content of support, the reference [5] divides the entrepreneurship policy into venture capital support, entrepreneurial site support, tax and fee relief support, and other support. According to the reference [6], the current entrepreneurship policies of college students in China can be divided into four categories, which are the entrepreneurship education policy, the entrepreneurship training policy, the entrepreneurial finance policy, and the entrepreneurial service policy. At present, domestic scholars' research on entrepreneurial policies mainly focuses on how to build a scientific and reasonable policy system. After a systematic review of the development of entrepreneurial policies, the reference [7] summarizes the entrepreneurial policy system of college students into four dimensions, namely, entrepreneurial education policy, entrepreneurial financing policy, business support policy, and entrepreneurial environment policy. However, reference [8] suggests that a sound entrepreneurship policy system should cover entrepreneurship education, financial support, and other aspects, including entrepreneurship education and training policy, entrepreneurship promotion policy, entrepreneurial financing policy, and entrepreneurial environment policy. Based on the AHP, the references [9, 10] construct an evaluation index system for the implementation effect of entrepreneurship support policies, which is used to evaluate the implementation effect of entrepreneurship support policies. It is found that the implementation effects of the number of training bases, the average profit of entrepreneurial enterprises, and the impact of stimulating the entrepreneurial intention are in the medium level. At present, there are few references that combine big data technology with the innovation of college students' entrepreneurship precise support path, which needs further research.

Firstly, this paper introduces the overall framework of the model, and the basic framework of the model is determined. Considering the elements of entrepreneurial support policies, the evaluation index of this paper is determined. Based on big data technology, the innovation model of college students' entrepreneurial precise support path is created, in which the *K*-means algorithm is applied to the innovation model of college students' entrepreneurial precise support path. Finally, the model is experimentally analyzed, and the performance of the model is tested.

## 2. The Overall Framework of the Model

Encouraging and supporting college students' entrepreneurship has important practical significance to solve the current employment problem. By mining potential entrepreneurial information resources, the big data analysis can not only bring more accurate judgment to college students' entrepreneurial path selection, but also help them grasp better entrepreneurial opportunities. From the perspective of big data technology, this paper expounds the basic principles of model design and analyzes the basic framework and implementation ideas of the research model.

### 2.1. The Basic Principles

The main purpose of the innovation model is to apply big data to the analysis of the accurate support path of college students' entrepreneurship, so as to improve the policy's practicability by understanding the opinions and opinions of college students on the entrepreneurship support policy. The overall structure and framework design of the model will directly affect the practicability of the model. In order to design a qualified innovation model, the following three requirements need to be met, as shown in Figure 1.

The scientific principle requires that researchers should always adhere to the principle of seeking truth from facts. The established evaluation index system should be able to reflect all aspects of college students' entrepreneurship support policies in an all-round way. The indicators are independent of each other and there is no cross, and the concept, value, and weight of each index are based on scientific basis.

The systematic principle means that the index should not only reflect the overall characteristics of the object, but also carry out the top-level design on the whole, so that the levels of each evaluation index form a clear, logical, and complete structure. Although the evaluation indexes are related to each other, there are clear boundaries and levels between each other.

The conciseness means that the index is intelligible and the evaluation index system should avoid tedious and complicated. When the evaluation index system is too cumbersome, the evaluation activities are often inconvenient to carry out, and the evaluators may have deviation in understanding the indicators, which has adverse impact on the final evaluation results. In order to avoid the above situation, when designing the evaluation index system, all levels of indicators should be concise to avoid duplication and tedious phenomenon, so as to ensure the scientific and reliable evaluation.

### 2.2. The Overall Framework

Based on big data analysis, this paper creates an innovation model of precise support path for college students' entrepreneurship. The model is mainly divided into five modules, which are the data collection, the data preprocessing, the model building, the operation model, and the result display, and the specific process is shown in Figure 2. The entrepreneurship support policy consists of several policy elements, which together constitute the dimensions of entrepreneurship support policy. Through the systematic review of domestic and foreign research, this paper divides the policy system of college students' entrepreneurship support into entrepreneurship education policy, entrepreneurship financing policy, business support policy, and entrepreneurial environment policy, and the entrepreneurship support policy of college students is analyzed.

The purpose of entrepreneurship education policy is to improve the theoretical literacy and cultivate their practical ability, in which a series of compulsory courses and lectures on entrepreneurship are offered to encourage college students to independently establish high-tech enterprises. The entrepreneurial financing policy is formulated by the government to ensure that college students' entrepreneurs obtain entrepreneurial funds, which can alleviate and alleviate the pressure of funds on entrepreneurship to a certain extent. The business support policy is to ensure the smooth development of entrepreneurial activities, whose goal is to reduce the resistances and reduce the cost of entrepreneurship through relevant policy tools. The entrepreneurial environment policy provides strong support for entrepreneurs to carry out entrepreneurial activities, which covers rich contents, such as the cultivation of entrepreneurial platform and the support of venture capital.

## 3. Innovation Model of Entrepreneurial Accurate Support Path Based on Big Data

Based on big data technology, this paper builds an innovation model of precise support path for college students' entrepreneurship. Before the specific feature analysis and construction, the data need to be preprocessed firstly. In this paper, the *K*-means algorithm is applied to the innovation model, and the evaluation criteria of the algorithm are introduced.

### 3.1. Innovation Model of Entrepreneurial Precise Support Path Based on *K*-Means

The clustering analysis is to solve the problem of data classification with arbitrary cluster shape, which is an unsupervised learning process to find similar element sets in data sets. According to the similarity of data, the clustering analysis can be divided into four categories: one is the clustering based on partition clustering, one is the clustering based on hierarchical, one is the clustering based on density, and the other is the clustering based on graph. The most representative algorithm is *K*-means clustering algorithm, which is sensitive to noise data in data sets. After comprehensive comparison of various algorithms, the *K*-means algorithm is finally selected for the model in this paper. If you want to use *K*-means algorithm, it is necessary to process noise data more strictly in the process of preprocessing, and it can also be improved in the process of actual analysis.

The *K*-means algorithm is a classical clustering algorithm based on partition, which has the advantages of easy to understand. The *K*-means algorithm gradually improves the clustering effect according to the characteristics of iterative method, which has been widely used in many researches, and many researchers have optimized it. The basic principle of *K*-means algorithm includes two main steps, and *k* objects need to be selected arbitrarily firstly, in which each object is a cluster centroid. For each remaining object, the corresponding distance formula can be used to calculate the distance between it and each centroid, and it is assigned to the cluster of centroids with the shortest distance. Then, the new centroid of each cluster can be obtained according to the average formula, and the above steps can be repeated until the criterion function converges. The model of college students' entrepreneurial precise support path and clustering algorithm is very realistic, so this paper chooses to use clustering algorithm to study the precise support path of college students' entrepreneurship.

The goal of clustering algorithm is generally expressed by objective function, the similarity of *K*-means algorithm is determined by Euclidean distance, and the quality of clustering is judged by the sum of squares of errors. For a data set with *n* data objects, the SSE of the algorithm is shown in the following formula, where SSE represents the intracluster error variance.

(1) $$\begin{array}{c} \text{SSE}=\overset{K}{\underset{k=1}{\sum }}\underset{X_{i}\in C_{\text{k}}}{\sum }{\left\|X_{i}-C_{k}\right\|}^{2}, \end{array}$$

where *X*_*i*_ represents the data set and *C*_*k*_ represents the category set after clustering analysis.

*c*_*k*_ is defined as the center point of cluster *C*_*k*_, and its calculation is shown in

(2) $$\begin{array}{c} c_{k}=\frac{\sum_{X_{i}\in C_{k}}X_{i}}{\left|C_{k}\right|}. \end{array}$$

By using the idea of greedy algorithm, the *K*-means algorithm modifies the clustering results through continuous, whose ultimate goal is to find the minimum clustering results, and the minimum SSE needs to be solved by the optimization problem. In the calculation process, there are mainly the following three ways to calculate the distance from the data object to the center of the data cluster, which are the Euclidean distance measurement formula, the Hamanton distance, and the included angle chord distance.

Because the basic ideas and principles of *K*-means algorithm and EM algorithm are the same, it is necessary to set the value of variables firstly; then, the above operation is repeated until it reaches the convergence standard. Therefore, the *K*-means algorithm is also an evolution of EM algorithm, and the specific steps are shown in Figure 3.

In the process of clustering analysis, the time requirement of *K*-means algorithm is directly proportional to the size of clustering data set. Among them, *i* represents the number of iterations at the time of convergence, *n* is the number of all data objects contained in all data sets required by clustering analysis, and *m* is the data attribute in the data set. However, most of the convergence process usually occurs in the early stage of clustering, so the value of *i* is generally small.

### 3.2. The Evaluation Criteria of the Model

The precision and recall are the best tools to measure the accuracy of prediction model, which is also used to judge the performance of the model in this article. By constantly adjusting the sampling mode and proportion, the accuracy of the model can be constantly improved. When there is inconsistency with *R* index, the model needs to be evaluated with *F* parameter, which is the weighted harmonic mean of precision and recall, as shown in

(3) $$\begin{array}{c} Z=\frac{T_{p}}{T_{p}+F_{p}}, \end{array}$$

(4) $$\begin{array}{c} R=\frac{T_{p}}{T_{p}+F_{N}}, \end{array}$$

(5) $$\begin{array}{c} F=\frac{\left(a^{2}+1\right)\text{ZR}}{a^{2}\left(Z+R\right)}, \end{array}$$

where *Z* represents the precision and *R* represents the recall. When the actual results are positive, *TP* represents that the prediction results are correct. When the actual result is negative, *FP* represents that the prediction result is correct. When the actual result is positive, *FN* represents the prediction result is wrong.

## 4. The Experimental Analysis and Results

### 4.1. The Data Acquisition

The data used in this paper is mainly obtained through the college students' entrepreneurship precision support path innovation questionnaire, which consists of two parts: one is the preface, and the other is the question. The preface of the questionnaire introduces the basic situation of the research and the questionnaire, which expounds the purpose of the survey to the respondents, and explains the problems needing attention in the process of filling in the questionnaire, so as to eliminate the possible doubts of the respondents in the process of filling in the questionnaire. The basic personal information mainly includes the gender, education background, major, participation in entrepreneurship competition, and school of the respondents, so as to ensure the universality and diversity of the survey samples. The implementation of college students' entrepreneurship support policy is the main part of the questionnaire, which is directly related to whether the questionnaire can accurately reflect the variables to be measured and the research problems. Starting from social benefits, policy understanding, policy utilization, policy satisfaction, policy coordination, and government service, the questionnaire sets up several measurement items for the evaluation index. In the process of this investigation, the evaluation method of the questionnaire is all measured by the Likert five scale; the higher the score is, the better the implementation effect of the entrepreneurial support policy of college students in Hebei Province is. On the contrary, it shows that there are some problems. The questionnaire used in this paper includes personal basic information and the implementation of college students' entrepreneurial support policies, which can better reflect the implementation effect of college students' entrepreneurial support policies.

The data preprocessing does not have a fixed process, which will change according to the different data sets. The general process can be divided into several aspects, one is the data cleaning, one is the data integration, one is the data conversion, and the other is the data specification.

The purpose of data cleaning is to delete the data irrelevant to the mining topic in the data set, and the missing values and outliers are processed to reduce noise data and eliminate the gap between data units [11]. The data integration is mainly to integrate different data on the data model, which can solve the conflict problem of data values. Through data integration, we can find and modify the inconsistent naming of data sources, and the repeated data in the data source can also be found. In the data set, the data of one attribute can be calculated by another attribute, which can result in data redundancy. The data redundancy refers to unnecessary repeated storage of data in memory, which will not only hinder the integrity of data in the database, but also cause a waste of storage space. For judging whether the attributes in the data source are redundant, there are relevant metrics, as shown in

(6) $$\begin{array}{c} \gamma_{A,B}=\frac{\sum \left(A-\bar{A}\right)\left(B-\bar{B}\right)}{\left(n-1\right)\sigma_{A}\sigma_{B}}, \end{array}$$

where *n* represents the number of tuples, $\bar{A}$ represents the average value of *A*, and *σ*_*A*_ and *σ*_*B*_ represent the standard deviation of *A* and *B*, respectively.

The specific calculation methods of *σ*_*A*_ and *σ*_*B*_ are shown in the following formulas:

(7) $$\begin{array}{c} \sigma_{A}=\sqrt{\frac{\sum {\left(A-\bar{A}\right)}^{2}}{n-1}}, \end{array}$$

(8) $$\begin{array}{c} \sigma_{B}=\sqrt{\frac{\sum {\left(B-\bar{B}\right)}^{2}}{n-1}}, \end{array}$$

where *γ*_*A*,*B*_ represents the data redundancy metric; if *γ*_*A*,*B*_ is greater than 0, there is a positive correlation between attribute *A* and attribute *B*, indicating that the value of *A* will increase with the increase of *B*. The larger the value of *γ*_*A*,*B*_ is, the greater the probability that one attribute contains another is. When the *γ*_*A*,*B*_ value is large enough, you can delete one of the attributes as redundant.

The data transformation is to transform the data in the data set into a storage form that is easy to carry out data mining, and the most common method is normalization. The normalization means that the attribute data is scaled in a certain scale so that it falls into a specific interval [12]. In addition, there are many ways to normalize, and the most commonly used method is zero mean normalization, which can be expressed by

(9) $$\begin{array}{c} v^{\prime }=\frac{v-\bar{A}}{\sigma_{A}}, \end{array}$$

where $\bar{A}$ represents the average of *A* and *σ*_*A*_ represents the standard deviation of *A*.

### 4.2. The Optimization of Sampling Mode

The training set of the model is sampled without sampling. By increasing the proportion of positive samples, this paper compares the influence of different up sampling proportion on prediction accuracy, so as to select the optimal sampling method. In this paper, six different samples are selected. The sample 1 is nonsampling mode; the samples 2, 3, 4, and 5 are up sampling; the percentage of positive samples is 20%, 40%, 60%, and 80%, respectively; and the sample 6 is a traditional statistical method. The accuracy of prediction under different sampling rates is shown in Figure 4. As can be seen from Figure 4, the recall and precision without sampling can reach 98.231% and 39.542%, respectively, which are better than other sampling methods. Therefore, we use the nonsampling method for modeling in this paper.

### 4.3. The Computational Complexity

The performance of the algorithm has a great impact on the model, this paper compares the operation time of the traditional algorithm and the *K*-means, and the results are shown in Figure 5. It can be seen that the operation time of the traditional algorithm is about 0.426 seconds, while that of the *K*-means algorithm is only 0.245 seconds, which is about half of the operation time of the traditional algorithm. The traditional algorithm has a high computational complexity, and the operation time of *K*-means algorithm is far less than the traditional algorithm, which greatly reduces the computational complexity of the algorithm.

### 4.4. The Precision, Recall, and *F* Parameter of the Model

The precision reflects the correct proportion of the model to each category, that is, the accuracy of the model in judging each category. The recall can reflect the sensitivity of the classification model to each category of data set, and *F* parameter can measure the comprehensive performance of the model on two indexes. In order to verify the model, the model using the traditional algorithm is set as the control group, and the *K*-means algorithm is set as the experimental group, and the results are shown in Figure 6.

Compared with the traditional algorithm, the *K*-means algorithm has better performance in improving precision, recall, and F parameter. In different samples, the precision of the two methods is 80.071% and 87.788%, respectively, and the precision of *K*-means algorithm is improved by 7.721% compared with the traditional algorithm. Similarly, the recall of *K*-means algorithm is improved by 9.542% compared with the traditional algorithm. In different samples, the *F* parameter of *K*-means algorithm can reach above 0.79, which indicates that the *K*-means algorithm can accurately predict the support path of college students' entrepreneurship.

## 5. Conclusion

Firstly, the basic principles of the innovation model for college students' entrepreneurial support path are analyzed, and the overall process of the model is determined. Then, the innovation model that is based on big data is established, in which the *K*-means is applied to the analysis of accurate support for entrepreneurship. Finally, the experimental results show that the *K*-means can greatly reduce the computational complexity, the precision of the *K*-means algorithm increases by 7.72%, and the recall increases by 9.54% compared with the traditional algorithm. In different types of samples, the *F* parameters of *K*-means algorithm can reach more than 0.79, which indicate that *K*-means algorithm can accurately predict entrepreneurial support path. The model is of great significance in improving the feasibility of college students' entrepreneurial support policy.

## Figures and Tables

**Figure 1:** The basic principles of model design.

**Figure 2:** The specific process of the model.

**Figure 3:** The flow chart of *K*-means algorithm.

**Figure 4:** The optimization of sampling mode.

**Figure 5:** The computational complexity.

**Figure 6:** The evaluation index of the model.

## Data Availability

The data set can be accessed upon request.
